# Principal Component Research of the Teaching Model Based on Multimodal Neural Network Algorithm

**DOI:** 10.1155/2022/5888299

**Published:** 2022-06-29

**Authors:** Guang Yang, Xiaodong Liang, Shanshan Deng, Xiao Chen

**Affiliations:** Hebei University of Chinese Medicine, Shijiazhuang, Hebei 050200, China

## Abstract

With the deepening and improvement of the contemporary English educating reform, the lookup on the satisfactory English training has attracted greater and extra attention. The key to enhance the English training is to enhance good teaching, and English teaching model is the key measure to enhance good schooling and teaching. Based on a single neural network, it can solely describe the randomness and irregularity of English education quality and cannot describe the whole exchange traits of English education model, which makes the impact deviation of teaching model larger. Based on the in-depth learning of the contemporary state of affairs and traits of English education model, blended with the traits of neural network, this paper constructs an English teaching model primarily based on multimodal neural network algorithm. The experimental results show that the convergence speed of multimodal neural network model is 76% higher than that of single network model, the sum of squares of average error is 79%, and the average evaluation accuracy is 13.99% and 6.42% higher than that of convolution neural network model and radial basis function neural network model, respectively. It is demonstrated that the multimodal neural network model does not accelerate the convergence speed of the network or improve the prediction accuracy of the model and can quickly realize the ability of global optimization. It shows the effectiveness and accuracy of using multimodal neural network algorithm to model English teaching quality and provides a feasible solution for teaching quality model.

## 1. Introduction

Deepening teaching reform and improving teaching quality are directly related to the quality of talent training. Fantastic teaching is the lifeline of the survival and improvement of greater education. The core mission of greater schooling is intelligence training, and the essential project of Genius education is teaching. The key to reform and development is to improve teaching quality. Teachers' study room teaching great assessment gadget is a key hyperlink to make sure the lecture room teaching is pleasant. A necessary measure to always enhance teaching administration and first-rate teaching is to set up a scientific teaching best comparison system. At present, school room teaching is nonetheless the important body, so enhancing the fine lecture room education has emerged as the principal task. The wonderful display of the classroom is essential to the beauty of education. Fantastic teaching is the basis of survival and development. The enchantment of first-rate education needs to be realized by means of strengthening the administration of educating units. Specific to every major, it is to pay interest to the fantastic curriculum construction, and the most primary key factor is that instructors must instruct every route they are accountable for. However, as for the modern-day assessment of curriculum education model, the giant majority of the strategies used are primarily based on a massive quantity of facts acquired from the questionnaire, using the weight formulated by experts in advance and the method of comprehensive scoring to obtain the evaluation results. This method has obvious subjectivity, and the experience stored in the expert brain is not conducive to dissemination and sharing. The use of manual calculation method will also seriously reduce the efficiency of evaluation.

In latest years, as a new technology, neural network has proven exceptional benefits in sample cognizance and classification, cognizance filtering, computerized control, prediction, and so on due to its fundamental traits such as nonlinear mapping, gaining knowledge of classification, and real-time optimization. Various neural networks can describe the randomness and irregularity of English teaching quality; however, due to the fact that a single machine cannot describe the whole trade traits of English educating model, the deviation of teaching great assessment is occasionally giant [1]. Therefore, some students put in advance the teaching brilliant distinction system of combined technology, which combines a couple of single utilized sciences together, makes use of their advantages to overcome their respective defects, determines the weight, and then constructs guided top-notch evaluation based on weights, and obtains an increased accuracy of excellent teaching evaluation of a single device [2]. The utility of multimodal neural network presents a new way for excellent teaching evaluation. Through nonstop process of gaining knowledge and training, multimodal neural network can locate its regularity from a giant wide variety of complex records of unknown modes. In particular, it can manner any kind of data, utterly proceed any complicated nonlinear relationship, simulate nonlinear processes, successfully clear up the hassle of nonlinear complete comparison, and limit the effect of human elements on decision-making results, which is unmatched by way of many common strategies [3]. Therefore, introducing the principle of multimodal neural network into the education first-rate assessment gadget no longer solely solves the issues of qualitative and quantitative warning signs in the complete contrast index system and overcomes the issues of organizing complicated mathematical fashions and mathematical analytical expressions in the ordinary assessment process, but it additionally avoids the direct impact of human elements on the assessment results, making the contrast more correct and effective. The education model set up with the aid of the idea of multimodal neural network is a high-quality technique for teaching first-class evaluation.

In this paper, the multimodal neural neighborhood algorithm is used to set up the English teaching model. Firstly, a scientific and real looking assessment index device is formulated, and then the dimension of the contrast index is decreased via the usage of the increased important element evaluation method. Then, the neural network assessment model of best teaching is determined, and the multimodal neural network algorithm is chosen to educate the sample data, gain the contrast results, and then affirm the verification data. The experimental results show that the convergence speed of multimodal neural network model is 76% higher than that of single network model, the sum of squares of average error is 79%, and the average evaluation accuracy is 13.99% and 6.42% higher than that of convolution neural network model and radial basis function neural network model, respectively.

Through multimodal neural network, we fairly consider the education quality, overcome the direct impact of human elements on the assessment results, and supply significant reference fee for the lookup of best teaching evaluation. The chapters and contents of this paper are organized as follows: Section 1 is the introduction, which presents the historical past and value of the research. Relevant work is mentioned in Section two. Section three introduces the applicable theories of neural network. In Section 4, the educational strategies that go with the flow and effects of the teaching model are analyzed, and the accuracy is simulated.  Section 5 summarizes the work carried out in this paper and factors out the similarly looked up content.

## 2. Related Work

With the rapid development of information technology and network technology, artificial neural network is applied in various fields, and its prediction function is gradually excavated. The working efficiency of artificial neural network is millions of times higher than that of neurons in human brain. For those programmable problems with clear rules of operation or reasoning, typical laws, or general characteristics, we can achieve fast and efficient solutions [4]. Because of its advantages of logic operation and numerical calculation speed and accuracy, it provides human beings with scientific and technological means to realize automation and intelligence in many aspects. However, its operation mechanism and structure mode still belong to the traditional logic operation rules, which cannot reach or surpass human thinking in many aspects [5]. Scientists are additionally actively searching for new methods to resolve such problems. The in-depth learning of human intelligence-shaped model and statistics processing mechanism has promoted the improvement of human talent science and promoted the improvement of synthetic neural network and the lookup of Genius model. Through in-depth research, artificial neural network has made great progress. After a long period of initial and low points, it finally ushered in the peak of the development of artificial neural network [6]. Through the improvement and perfection of its function and structure by researchers over the years, its operation mechanism has gradually matured, its application field has been continuously extended, and many problems in the industry have been solved. It shows that it has great potential, and its remarkable achievements have been widely recognized. The prediction of the development of things can be realized by artificial neural network modelling, which will save the research time required for the actual verification results.

Governments and firms in many nations have invested a lot of human and cloth assets in neural network research. Try to take the lead in this new discipline field, and carry out exploration, research, and development from the aspects of application, theory, model, algorithm, and time limit [7]. With the deepening of research, researchers have always launched neural network fashions and simulation programs, posted a giant wide variety of scientific lookup papers, and the lookup in exclusive industries has additionally been posted in the newspapers, which suggests that a state of affair of competition amongst a hundred faculties of idea has progressively shaped in the subject of neural network lookup [8].

At present, it is impossible to give a more authoritative definition of artificial neural network, but it can be understood as using the working mode of bionic brain to simulate human brain to realize some functions, extracting some “neurons” and connecting them in a special way to form a topology [9]. It also has some characteristics of the human brain, such as strong fault tolerance. Because the information is stored in the whole network, rather than being limited to a specific area, the efficiency of processing information as a single neuron may be slow, but the whole neural system can quickly respond to specific information processing, and batch parallel processing of information can also be realized in this process [10]. The neural gadget can additionally deal with issues such as unsure reasoning rules, uncertain records historical past, or complicated environmental information, because the artificial neural machine has the qualities of sturdy adaptability, self-learning, and self-organization [11].

## 3. Related Theories of Neural Network

### 3.1. Convolutional Neural Network

Convolutional neural network is one of the representative algorithms of artificial neural network. It is named after its unique convolution operation. It belongs to the classical deep feedforward neural network in deep learning. Convolution neural network has the capability of representation learning, can maintain the hierarchical structure of the original data and transform and judge the input information accordingly, and has translation invariance to the characteristic information, so it is also called translation invariant artificial neural network [12]. Convolution kernel operator extracts the features of matrix data by sliding window movement, which is very suitable for image information processing. The common CNN structure is shown in Figure 1.

Convolutional layers are the core components of convolutional neural networks, which have local connections and weight sharing features [13]. The neurons in the identical characteristic map of the convolutional layer extract nearby elements at specific positions in the characteristic map of the preceding layer, whilst for a single neuron, the extracted aspects are the neighborhood elements of the identical role in countless one-of-a-kind function maps of the preceding layer [14]. What the convolutional layer accomplishes is that one or more attribute maps of the previous layer are used as entry to function a convolution operation with one or more convolution kernels to generate one or more outputs.

The convolutional neural network predicts and classifies the multiclassification problem at the end of the network layer and changes the output of the last neuron into the form of probability, so that the model can output a probability distribution at the end [15], only when the calculation results of the output layer are converted into probability models through SoftMax function for output. The SoftMax function formula is

(1) $$\begin{array}{c} H_{D}\left(\alpha^{\left(i\right)}\right)=\frac{{\left[e^{D_{1}^{T}\alpha \left(i\right)}\right]}^{T}*{\left[e^{D_{2}^{T}\alpha \left(i\right)}\right]}^{T}*\cdots *{\left[e^{D_{51}^{T}\alpha \left(i\right)}\right]}^{T}}{\sum_{j=1}^{51}e^{D_{j}^{T}\alpha \left(i\right)}}. \end{array}$$

The softmax function converts the calculation results of all network nodes in the output layer into a probability distribution and at the same time makes the influence of the features on the probability multiplicative [16]. During coaching new release manner of the network model, the general error of the network is calculated when backpropagating and correcting increase comfort and velocity and can smoothly apply the chain rule to update the weights [17]. The loss function of this model is

(2) $$\begin{array}{c} \xi \left(\sigma ,\tau \right)=\frac{50\lambda \sum_{i=1}^{51}\sum_{j=0}^{2048}\sigma_{i,j}^{2}-\sum_{i=1}^{100}\sum_{j=1}^{51}\left(\left\{\beta^{\left(i\right)}=j\right\}\right)\ln\left(e^{D_{j}^{T}\alpha \left(i\right)}/\sum_{i=1}^{51}D_{\ell }^{T}\alpha \left(i\right)\right)}{100}. \end{array}$$

In order to ensure that the data maintains the same distribution before entering the convolutional layer to reduce the impact of related factors on the training results, a data normalization operation is added before the second convolutional layer Conv-2 and the fourth convolutional layer Conv-4 [18]. This paper adopts batch normalization operation. The normalization operation is a very effective data processing method, which can make the network more robust, accept a higher learning rate, and at the same time reduce the dependence on accurate initialization and reduce overfitting:

(3) $$\begin{array}{c} \sigma_{ij}^{\left(\ell \right)}=\frac{-\partial \xi \left(\sigma ,\tau \right)+\sigma_{ij}^{\left(\ell \right)}\cdot \partial \sigma_{ij}^{\left(\ell \right)}}{\partial \sigma_{ij}^{\left(\ell \right)}},\\ \tau_{i}^{\left(\ell \right)}=\frac{-\partial \xi \left(\sigma ,\tau \right)+\sigma_{i}^{\left(\ell \right)}\cdot \partial \sigma_{i}^{\left(\ell \right)}}{\partial \sigma_{i}^{\left(\ell \right)}}, \end{array}$$

where *σ*_*ij*_^(*ℓ*)^ represents the weight parameter of the connection between the *i*th neuron of layer *ℓ*+1 and the *j*-th neuron of layer and *τ*_*i*_^(*ℓ*)^ represents the bias term of the *i*th neuron of layer *ℓ*+1.

Since the image size of the dataset is different from the standard input image size of the model, it is necessary to scale and transform the image size of the dataset. In order to ensure that the image quality is less damaged after scaling the image size, this paper uses a bicubic interpolation scaling algorithm to the size of the image that is standardized, which can effectively ensure the integrity of the image feature information. The image size is not much different from the standard input size of the model [19]. Under this premise, scaling the image to the corresponding size will only have a small impact on the original image feature information:

(4) $$\begin{array}{c} \frac{\partial \xi \left(\sigma ,\tau \right)}{\partial \sigma_{ij}^{\left(\ell \right)}}=\varsigma_{i}^{\left(\ell \right)}\alpha_{j}^{\left(\ell -1\right)},\\ \frac{\partial \xi \left(\sigma ,\tau \right)}{\partial \tau_{i}^{\left(\ell \right)}}=\varsigma_{i}^{\left(\ell \right)}. \end{array}$$

### 3.2. Artificial Neural Network

The thought of artificial neural network originated from learning about talent neural network through biologists, from which the working precept of its neurons used to be found, and a perceptron model was once proposed from a mathematical factor of view to summarize it. In the in-depth lookup and exploration of intelligence structure, it is discovered that, below the stimulation of the backyard world, the intelligence has a complicated response gadget between its inner neurons and inside the worried system, simulates the working precept of the brain, and constructs a multilevel perceptron mathematical model, additionally recognized as synthetic neural network, which can perform easy classification processing tasks [20]. Because of its advantages, the impact of synthetic neural network model in many lookup fields is tons higher than that of the regular algorithm. It has precise software fee and enterprise prospects and has attracted the pastime and interest of students in a number neighborhood [21].

In the synthetic neural network model, every network layer is organized in parallel to manner and calculate statistics synchronously. At the same time, it has accurate fault tolerance, can fuse and analyze the attribute statistics of records by itself, and has robust self-learning ability. Finally, it determines the most splendid model parameters, which has excellent adaptability and generalization for new statistics information. Its primary unit is neurons [22]. There are elaborate connection relationships between neurons, and the information between neighborhood layers is rather nonlinear. Therefore, it can mine a quantity hidden logical relationships between factors and whole elaborate processing and calculation. It is a large-scale nonlinear characteristic turning into system. As a precis computing system, its essence is to combine the easy ideas of human natural neural neighborhood with rich mathematical theories and methods and use computing tools to set up mathematical fashions [23]. Therefore, artificial neural neighborhood moreover is conveniently getting to be aware of ability, judgment plausible and prediction functionality the same as the human brain, and its cross-perception calculus principle has been extended to multidisciplinary theoretical lookup systems.

Any unit node in the synthetic neural network can raise out nonlinear mapping and processing on the entered data and raise out mathematical degree transformation and similarly calculation on exceptional sorts of tasks, such as language, sound, image, text, signal, and different types of records data [24]. The fine mixture of records and extraordinary processing strategies of distinct statistics is expressed in this complicated connection network. The neural network is no longer bendy and adaptable to the standard neural network [25]. In terms of statistics processing methods, it imitates the fashion of the intelligence and has magnificent portability and generalization ability. In essence, it is a multilevel and dispensed statistics processing system. In terms of structure, it fashions the connection and mixture of intelligence worried machine devices to a sure extent and correctly integrates a range of advantages, so as to assemble such a complicated large-scale built-in gadget of information processing, analysis, calculation, and prediction [26].

### 3.3. Radial Basis Function Neural Network

RBF neural network consists of three layers: input layer, hidden layer, and output layer. There is no weight connection between the input layer and the hidden layer, and the input vector is at once mapped to the hidden layer. The mapping from input layer to hidden layer is nonlinear; that is, the transformation characteristic of hidden layer is a nonlinear function. There are connection weights between the hidden layer and the output layer. The mapping from the hidden layer to the output layer is linear; that is, the output of the complete network is the linear weighted sum of the output consequences of the hidden layer [27]. The imperative big difference between RBF neural neighborhood and exclusive feedforward neural networks is the hidden layer. The “basis” of the hidden layer residence adopts the radial groundwork function, so that as quickly as the center of the radial basis attribute of each and every hidden layer node is determined, the input vector can be mapped to the hidden layer location barring weight connection. The range of neural networks is mirrored now not only in the network model decided through the quantity of hidden layer nodes, but also in the chosen radial groundwork function. In terms of structure, RBF neural network has easy topology and easy and clear mastering and coaching process. It takes the radial foundation characteristic as the activation function [28]. Only when the input sign is shut to the center of the radial foundation function, the hidden layer node can produce a giant output. The topology of RBF neural network is proven in Figure 2.

When the hidden layer node of the neural network chooses to use the radial groundwork characteristic as the activation function, it constitutes the radial foundation feature neural network. The simple notion of its layout is the cowl theorem, that is, undertaking the low-dimensional linear inseparable information into a new space, making the information linearly separable in the new area through sensible plan and selection, and then using the linear aspect to deal with the problem; for example, the expected output price is bought by using linear weighting in the output layer. There are complicated connection relationships between neurons, and the facts between network layers are enormously nonlinear. Therefore, it can mine quite a few hidden logical relationships between factors and perform whole elaborate processing and calculation. It is a large-scale nonlinear function turning into system. As a precis computing system, its essence is to combine the easy standards of human natural neural neighborhood with rich mathematical theories and methods and use computing gear to set up mathematical models.

It can additionally be considered that the parameters of RBF neural network needed to be adjusted encompass 4 parts: central position, width, extent of foundation characteristic, and weight of output unit. Firstly, mixed with a range of neural network coaching methods, decide the central role of the network and different free variables in the activation function, and then the linear mapping relationship of the output layer can be mixed with the least rectangular technique to achieve the weight matrix of the output layer by means of fixing the matrix equation. Therefore, in the network training, the education of the center role and width of the foundation characteristic is the key section of the design.

## 4. Analysis and Results

### 4.1. Analysis of Prediction Results of Teaching Model

Since the indications of the education first-class comparison device set up in this paper are fantastic indicators, the records translation steps are omitted. The preliminary assessment outcomes of the education great assessment warning signs are decided in accordance with the steps of the direct cost approach described, as shown in Figure 3.

The switch characteristic used in the output layer of neural network is *S*-function, and the fee variable of *S*-shaped characteristic is constrained to (0, 1); that is, the output variable of neural network is (0, 1), so the output of education records needs to be normalized to the interval of [0, 1]. The initial evaluation value range of teaching quality determined by the direct value method is (0, 1), so the data standardization is carried out again. Finally, 1000 groups of data are determined to participate in the experiment, of which 900 groups are used to train the model so as to obtain the optimal BP neural network structure, and the remaining 100 groups of data are used for testing. Some test data are shown in Figure 4 to test the performance of the model.

Among them, 1 to 18 columns of every crew of samples, namely, the records of 18 secondary indicators contained in the 5 fundamental indicators of teachers' quality, education attitude, teaching content, teaching technique, and education effect, are used as the input price of the network test, namely, columns *x*_1_, *x*_2_, *x*_3_,…, *x*_17_ and *x*_18_ of every crew of data. The secondary indicator rating is the input information of the neural network, and the preliminary contrast end result based totally on the direct fee technique is the output goal of the network. The first crew of input samples *P* = (0.90, 0.87, 0.86,…, 0.94, 0.87), and the output is *F*1 = 0.88. By analogy, proceed to learn, reap an ideal model, enter the ranking facts of teaching excellent distinction warning signs and indicators from crew 901 to crew 1000, and predict and output the teaching brilliant evaluation results through neural network. Through the verification and checking out of the model, it can be noted that the model can make a nicely timed and scientific evaluation of teaching quality. The prediction results of the teaching quality evaluation model are shown in Figure 5.

### 4.2. Convergence Accuracy Analysis of the Model

Comparing the implied rectangular error curve, it is observed that the implied rectangular error of the first 30 iterations of the single neural network algorithm decreases rapidly, the thirty first to eightieth iterations are slow and converge after 87 iterations, and the suggested rectangular error converges at 8.6066*e* − 8. The convergence pace of technology 93*e* − 2 neural network is faster than that of technology 389*e* − 2 neural network, and the convergence pace of technology 389*e* − 12 neural network occurs to a sure extent. The convergence speed is more, and the modal neural network model is extended through 79.31%, and the convergence accuracy is almost doubled. It suggests that the multimodal neural network model cannot solely speed up the convergence pace of the network; however, it additionally enhances the prediction accuracy of the model. Comparison of convergence speed of different neural network algorithms is shown in Figure 6.

Further evaluating the alternate of the rectangular sum of error of the single neural network algorithm and the rectangular sum of error of the multimodal neural network algorithm, it can be viewed from Figure 7 that the common rectangular sum of error and the minimal rectangular sum of error of the single neural network algorithm converge rapidly earlier than the tenth generation, and the convergence pace of the tenth to twenty-fifth era is slow. Finally, it converges to the twenty-fifth iteration, and the rectangular sum of error is secure at about 0.9. The multimodal neural network algorithm converges after solely six iterations. The sum of error squares of the network is stable, the sum of error squares converges to 0.19, the convergence pace is accelerated by 76%, and the common sum of error squares is decreased by 79%. After comparison, it can be viewed that the multimodal neural network algorithm can shortly understand world optimization.

Figure 8 indicates that the common fitness and best fitness of a single neural network algorithm converge quicker and earlier than the twentieth generation, slowly from the fortieth to sixtieth generation, attain a consistent country after sixty-seven iterations, and ultimately stabilize at 0.84. The fitness of the multimodal neural network model converges to the twentieth iteration, and the fitness price is secure at 1.44. After comparison, it can be considered that the multiplied model has excessive adaptability and has been optimized to a sure extent.

The contrast outcomes of common contrast accuracy are proven in Figure 9. The common assessment accuracy of convolution neural network model for a hundred businesses of records is 84.26%, that of radial foundation characteristic neural network model is 91.83%, and that of multimodal neural network algorithm is 98.35%, which is 13.99% and 6.42% greater than convolution neural network and radial foundation characteristic neural network, respectively.

## 5. Conclusion

We aimed at discussing the negative aspects that a single neural network can solely describe the randomness and irregularity of first-rate English teaching and cannot describe the whole trade traits of English education model, which makes the impact deviation of teaching model surprisingly massive and the universality of educating model poor, and enhancing the education of schools and universities, primarily based on the in-depth knowledge of the modern state of affairs and traits of English teaching model, blended with the traits of neural network. This paper constructs an English education model primarily based on multimodal neural network algorithm, selects multimodal neural network algorithm to educate the pattern data, obtains the contrast results, and then verifies the verification data. Experimental data show that the multimodal neural neighborhood has a faster convergence effect and more accurate prediction accuracy in English teaching mode search. It will expand the effectiveness and accuracy of English teaching exquisite modelling and present a feasible response for teaching first-rate modelling. Teaching evaluation is a very elaborate and fuzzy nonlinear process, even though this paper analyzes and improves the issues of English teaching model, it is hoped that some sensible issues can be studied in a similar fashion in the future.

## Figures and Tables

**Figure 1:** Basic process of logistics distribution.

**Figure 2:** Structure of RBF neural network.

**Figure 3:** Result data of initial evaluation.

**Figure 4:** Test input data after normalization.

**Figure 5:** Prediction results of teaching quality evaluation model. (a) Evaluation value of different samples. (b) Predictive value of multimodal neural network algorithm.

**Figure 6:** Comparison of convergence speed of different neural network algorithms. (a) Mean square error of single neutral network algorithm. (b) Mean square error of multimodal neutral network algorithm.

**Figure 7:** Comparison of convergence errors of different neural network algorithms. (a) Sum of squares of single neutral network error. (b) Sum of squares of error of multimodal neutral network.

**Figure 8:** Comparison of fitness of different neural network algorithms. (a) Fitness of single neutral network algorithm. (b) Fitness of multimodal neutral network algorithm.

**Figure 9:** Performance comparison of different neural network models.

## Data Availability

All data, models, and codes generated or used during the study are presented in the submitted paper.
